This article has been retracted.

# The Choice of Anesthetic Drugs in Outpatient Hysteroscopic Surgery: A Systematic Review and Network Meta-Analysis

**DOI:** 10.1155/2022/2408685

**Published:** 2022-09-21

**Authors:** Shengnan Li, Bin Wu, Bibo Peng, Qian Zhang, Hongdan Zhao, Kun Hou, Lina An

**Affiliations:** ^1^Outpatient Department, Third Medical Center of Chinese PLA General Hospital, 69 Yongding Road, Haidian District, Beijing 100039, China; ^2^Department of Anesthesiology, Third Medical Center of Chinese PLA General Hospital, 69 Yongding Road, Haidian District, Beijing 100039, China

## Abstract

**Objective:**

Hysteroscopy is a minimally invasive gynecologic technique that is widely practiced in outpatient procedures. The choice of anesthesia is a key factor for the surgical outcome and postoperative recovery. This study was conducted to assess the effects of different anesthetic modalities based on dexmedetomidine in outpatient hysteroscopic surgery anesthesia.

**Methods:**

We did a systematic review and network meta-analysis of outpatient hysteroscopic surgery anesthesia. We searched Pubmed, Embase, and Cochrane-Library from database inception to December 31, 2021. Duplicate literature was excluded and screened separately for initial screening at three tiers: article title, abstract, and full text before deciding whether to include in this study against the above criteria. Results after analysis of categorical variables were expressed as ORR Ratio (95% CI) and continuous variables were expressed as Mean Difference (95% CI). Data collation and analyses were performed using the gemtc package in the R language.

**Results:**

Four trials were finally included with data for 301 participants, three anesthetic drugs, and five anesthetic modalities. A fixed-effects model was used for the different anesthesia modalities without significant heterogeneity (all I2<20%) in the analysis of adverse events (AEs), the incidence of respiratory depression, operative time, and time in the post-anesthesia care unit (PACU). Remimazolam tosylate was associated with a lower incidence of AEs versus dexmedetomidine, and significant differences between dexmedetomidine and propofol were absent. Propofol and various doses of remimazolam tosylate resulted in a lower incidence of respiratory depression versus dexmedetomidine, with an absence of differences between propofol and dexmedetomidine. The operative time for different anesthetic modalities was, in descending order, dexmedetomidine < remimazolam tosylate (0.60 mg/kg/h <0.48 mg/kg/h) < propofol < remimazolam tosylate (1.00 mg/kg/h), despite the absence of intergroup differences. Propofol was associated with a longer time in PACU versus dexmedetomidine and remimazolam tosylate (1.00 mg/kg/h); those of dexmedetomidine and remimazolam tosylate (1.00 mg/kg/h) were similar. The time in PACU for different anesthetic modalities, in descending order, was dexmedetomidine < remimazolam tosylate (1.00 mg/kg/h) < propofol. Propofol was associated with a longer time in PACU versus dexmedetomidine and remimazolam tosylate.

**Conclusion:**

In outpatient hysteroscopic surgery anesthesia, dexmedetomidine was associated with a higher incidence of AEs and respiratory depression and a shorter operative time and time in PACU versus remimazolam tosylate and propofol. Remimazolam tosylate showed safety benefits with a similar duration of PACU stay versus dexmedetomidine. Therefore, the choice of anesthetic drugs in outpatient surgery requires consideration of the patient's conditions and preferences.

## 1. Introduction

Hysteroscopy provides a clear view of the changes in the uterine cavity to aid physicians for accurate diagnosis [1]. The use of hysteroscopy for precise and standardized diagnosis and treatment of uterine cavity diseases is currently widespread worldwide [2, 3]. Outpatient surgery is simple and accessible but also imposes higher requirements on the safety and efficiency of anesthetic drugs [4]. Short-acting anesthetics with reasonable drug combinations and doses are appreciated in outpatient hysteroscopic surgery with short preoperative preparation to facilitate postoperative recovery [5].

Dexmedetomidine is a relatively selective *α*2-adrenoceptor agonist that provides sedation and analgesia with a lesser dose and mild respiratory depression and is now extensively used in clinical practice [6, 7]. Dexmedetomidine may increase vagal tone, causing hypotension, bradycardia, and sinus arrest, which can be relieved by a slow infusion, and it can also reduce oxygen consumption and redistribution of coronary blood flow in nonischemic areas to provide benefit in ischemic heart disease [8]. Moreover, dexmedetomidine is characterized by good intraoperative arousal [9]. Dexmedetomidine, propofol, and remimazolam tosylate were all common anesthetic drugs in outpatient hysteroscopic surgery [10, 11]; however, the efficacy of the three drugs in outpatient hysteroscopic procedures is marginally studied.

Meta-analysis has been widely applied for disease study, including the outpatient surgeries [12, 13]. A previous meta-analysis indicated that intracervical and paracervical injections of local anesthetic significantly reduced the pain in women who received outpatient hysteroscopy, whereas transcervical and topical application did not [14]. These meta-analyses provide important guidance and evidences for clinical practice. Nevertheless, no study on choice of anesthetics for outpatient hysteroscopic surgery was recently conducted. Accordingly, this meta-analysis was carried out to compare the efficacy of dexmedetomidine, propofol, and remimazolam tosylate in outpatient hysteroscopic surgery anesthesia to provide a reference for clinical treatment.

## 2. Materials and Methods

### 2.1. Literature Search

A literature search was conducted on Pubmed, EMbase, and Cochrane-Library from database inception to December 31, 2021, using the search terms of ((hysteroscope [Title/Abstract]) or (uteroscope [Title/Abstract]) or (metroscope[Title/Abstract]) and ((Dexmedetomidine [Title/Abstract]) or (DEX [Title/Abstract])), without language filters for searching. References of the included literature were searched and retrospectively added to potentially missing studies whenever possible.

### 2.2. Inclusion and Exclusion Criteria

#### 2.2.1. Inclusion Criteria

The inclusion criteria are as follows: (1) study type is Randomized Comparison clinical Trial (RCT) or Clinical Trial; (2) study participants are patients who underwent outpatient hysteroscopic procedures with at least two of dexmedetomidine, propofol, or remimazolam tosylate used for anesthesia; (3) outcome measures included hemodynamic status, perioperative indicators (anesthesia time, total operative time, and awakening time); and (4) the study design was scientific and standardized, with clear grouping and interventions and complete documentation such as follow-up data.

#### 2.2.2. Exclusion Criteria

The exclusion criteria are as follows: (1) nonclinical studies, case reports, or secondary data analysis; (2) inability to extract relevant outcome indicators; and (3) inclusion of fewer than 15 participants in a single group.

### 2.3. Literature Screening

Retrieval of data was carried out by two investigators, and literature management was conducted using Endnote. Duplicate literature was excluded and screened separately for initial screening at three tiers: article title, abstract, and full text before deciding whether to include in this study against the above criteria. Quality assessment of the included literature using the Cochrane risk-of-bias tool, and the decision to include was made by a third investigator independently for discrepancies between the two investigators.

### 2.4. Data Extraction

The following data were extracted by two investigators independently from the included studies: first author's name, year of publication, subject type, number of subjects, treatment, study design, hemodynamic status, perioperative indicators (anesthesia time, operative time, and awakening time), anesthetic drug dosage, and postoperative adverse events. Postoperative adverse events, operative time, and time in PACU were considered meta-analysis main effect measures.

### 2.5. Statistical Analysis

Data collation and analyses were performed using the gemtc package in the R language. Postoperative adverse events data included sample size and case, and operative time and time in PACU data included mean value, std.dev, and sampleSize. The I2 test was used to evaluate the heterogeneity of the included studies. I2 = 0 and *P* > 0.1 for both subgroups indicated no heterogeneity in the included studies, and 50% > I2> 0 and *P* < 0.1 indicated mild heterogeneity. A fixed-effects model was used for all analyses. Results after analysis of categorical variables were expressed as ORR Ratio (95% CI) and of continuous variables were expressed as Mean Difference (95% CI).

## 3. Results

### 3.1. Eligible Literature

Of 400 original papers retrieved by an electronic search, 312 papers were excluded after literature abstracts reading and exclusion of case reports, abstracts, and reviews, and 58 papers were coarsely included. Following the reading of the full text, studies with duplicate reports and unspecified data were ruled out, and the final 4 pieces of literature were recruited. The four trials included 301 participants, 3 anesthetic drugs (dexmedetomidine, propofol, remimazolam tosylate [0.48 mg/kg/h, 0.60 mg/kg/h, 1.00 mg/kg/h]), and 5 treatment regimens. There were one 3-arm study of propofol versus remimazolam tosylate, 2 studies of propofol versus dexmedetomidine, and 1 study of remimazolam tosylate versus propofol. The 3-arm study (propofol, remimazolam tosylate 0.48 mg/kg/h, remimazolam tosylate 0.60 mg/kg/h) was converted into 2 two-arm studies (propofol vs. remimazolam tosylate 0.48 mg/kg/h. Propofol vs remimazolam tosylate0.60 mg/kg/h). The basic information of the included literature is shown in Table 1, the quality evaluation of the included literature is shown in Figure 1, and the network diagram of enrolled studies is shown in Figure 2.

### 3.2. Incidence of Adverse Events

Analysis of the incidence of postoperative adverse events was found in 3 studies, with an interstudy heterogeneity of I2 = 16% and no significant heterogeneity found between groups. A fixed-effects model was employed for analysis. Remimazolam tosylate was associated with a lower incidence of AEs versus dexmedetomidine, and significant differences between dexmedetomidine and propofol were absent. The incidence of AEs was, in descending order, remimazolam tosylate (0.48 mg/kg/h < 1.00 mg/kg/h < 0.60 mg/kg/h) < propofol < dexmedetomidine, without significant differences between groups (Figure 3).

### 3.3. Respiratory Depression

Three studies analyzed the incidence of respiratory depression, with an interstudy heterogeneity of I^2^ = 17% and no significant heterogeneity found between groups. A fixed-effects model was employed for analysis. Propofol and various doses of remimazolam tosylate resulted in a lower incidence of respiratory depression versus dexmedetomidine, with an absence of differences between propofol and dexmedetomidine. The incidence of respiratory depression for different anesthetic modalities was, in descending order, remimazolam tosylate (1.00 mg/kg/h < 0.60 mg/kg/h <0.48 mg/kg/h) < propofol < dexmedetomidine, without significant differences between groups (Figure 4).

### 3.4. Operative Time

Three studies analyzed operative time, with an interstudy heterogeneity of I^2^ = 12% and no significant heterogeneity found between groups. A fixed-effects model was employed for analysis. Propofol and different doses of remimazolam tosylate presented a longer operative time versus dexmedetomidine, without notable differences between dexmedetomidine and propofol. The operative time for different anesthetic modalities was, in descending order, dexmedetomidine < remimazolam tosylate (0.60 mg/kg/h <0.48 mg/kg/h) < propofol < remimazolam tosylate (1.00 mg/kg/h), despite the absence of intergroup differences (Figure 5).

### 3.5. Time in PACU

Three studies analyzed the time in PACU, with an interstudy heterogeneity of I^2^ = 12% and no significant heterogeneity found between groups. A fixed-effects model was employed for analysis. Propofol was associated with a longer time in PACU versus dexmedetomidine and remimazolam tosylate (1.00 mg/kg/h); those of dexmedetomidine and remimazolam tosylate (1.00 mg/kg/h) were similar. The time in PACU for different anesthetic modalities, in descending order, was dexmedetomidine < remimazolam tosylate (1.00 mg/kg/h) < propofol. (Figure 6).

## 4. Discussion

The results of this study showed that dexmedetomidine was associated with a higher incidence of adverse events and respiratory depression and a shorter operative time and time in PACU versus propofol and remimazolam tosylate. Hysteroscopy is an endoscopic examination that allows direct visualization of intrauterine lesions, provides a rapid and accurate diagnosis of most intrauterine diseases, and has become the diagnostic gold standard for assessing intrauterine lesions [15]. Hysteroscopic surgery is less invasive with fast recovery, which results in a better medical experience for the patients. However, higher demand for better anesthesia is presented by outpatient surgery due to short preoperative preparation and high postoperative awakening requirements. Thus, postoperative adverse events and postoperative recovery are major concerns in outpatient surgery [16]. Dexmedetomidine, propofol, and remimazolam tosylate are commonly used anesthetic drugs, but comparisons of their effects in adverse events and postoperative recovery have been marginally reported.

In the present study, propofol showed a promising safety profile but a prolonged stay of patients in PACU. Propofol is a short-acting intravenous anesthetic for the induction and maintenance of general anesthesia and is frequently used with epidural or spinal anesthesia, analgesics, inotropes, and inhalational anesthetics [17]. Propofol is associated with a rapid and smooth entry into anesthesia as evidenced by a sleep state within 40 seconds after intravenous administration and can also mitigate the negative emotions of patients. However, the poor analgesic effect of propofol may decrease intracranial pressure, cerebral oxygen consumption, and cerebral blood flows [18]. In addition, its suppressive effects on the respiratory and circulatory systems may result in temporary respiratory arrest or blood pressure reduction [19], which entails strict compliance with the doctors' advice. Furthermore, propofol may also elicit damage to the nervous system, digestive system, skin and its adnexa, nutritional metabolism disorders, and dependence, necessitating close postoperative monitoring [20].

Here, remimazolam tosylate presented a manageable safety and comparable length of stay in PACU of patients. Remimazolam tosylate is a new anesthetic sedative with rapid onset and breakdown, no significant respiratory or cardiovascular effects, and it is also metabolized by tissue esterases with inactive metabolites that can be antagonized by flumazenil, showing better anesthetic enrichments over midazolam and propofol [21]. Research has shown that remimazolam tosylate exhibited a time-dependent half-life independent of infusion time compared with dexmedetomidine and propofol and had a shorter awakening time than propofol in gastroscopic practices [22]. General anesthesia experiments showed a satisfactory sedation depth for both remimazolam tosylate and propofol, and its advantageous features in colonoscopy and general anesthesia demonstrate its great potential in postoperative sedation of outpatient hysteroscopic procedures [23].

## 5. Conclusion

In outpatient hysteroscopic surgery anesthesia, dexmedetomidine, was associated with a higher incidence of AEs and respiratory depression and a shorter operative time and time in PACU versus remimazolam tosylate and propofol. Remimazolam tosylate showed safety benefits with a similar duration of PACU stay versus dexmedetomidine. Therefore, the choice of anesthetic drugs in outpatient surgery requires consideration of the patient's conditions and preferences. Further research with more literatures should be performed in future study.

## Figures and Tables

**Figure 1:** Quality evaluation chart of enrolled literature.

**Figure 2:** Network diagram of enrolled studies.

**Figure 3:** Network meta-analysis of AEs compared with DEX.

**Figure 4:** Network meta-analysis of Respiratory depression compared with DEX.

**Figure 5:** Network meta-analysis of Operation time compared with DEX.

**Figure 6:** Network meta-analysis of PACU time compared with DEX.

**Table 1:** Basic information of the included literature.

Author	Year	Type	Total cases	Arm 1	Arm 2	Outcome
Zhang S [1]	2022	RCT	90	Propofol	Remimazolam Tosylate (0.48 mg/kg/h)	HR, MAP, SpO2, OAA/S, AEs
				Propofol	Remimazolam Tosylate (0.60 mg/kg/h)	HR, MAP, SpO2, OAA/S, AEs
Bingol TT [2]	2019	RCT	60	Dexmedetomidine	Propofol	VAS, HR, MAP, SpO2, SAS
Park S [3]	2020	RCT	69	Dexmedetomidine	Propofol	AEs, MAP, HR, SpO2, OAA/S
Zhang X [4]	2021	RCT	82	Remimazolam Tosylate (1.00 mg/kg/h)	Propofol	AEs, MAP, HR

## Data Availability

The datasets used during the present study are available from the corresponding author upon reasonable request.
